# Clinical Significance of Protective Motivation Intervention Nursing on Functional Recovery of Patients after Hip Arthroplasty

**DOI:** 10.1155/2022/4219131

**Published:** 2022-09-09

**Authors:** Xue Yuan, Fengqin Xu, Shou Lin Zhu, Lijuan Huo, Ying Chen

**Affiliations:** ^1^The First Affiliated Hospital of Kangda College of Nanjing Medical University/The First People's Hospital of Lianyungang Joint Surgery Nursing Unit, Lianyungang, Jiangsu 222000, China; ^2^The First Affiliated Hospital of Kangda College of Nanjing Medical University/The First People's Hospital of Lianyungang Nursing Department, Lianyungang, Jiangsu 222000, China

## Abstract

**Objective:**

To explore the clinical significance of protective motivation intervention nursing on functional recovery of patients after hip arthroplasty.

**Methods:**

Sixty patients after hip arthroplasty treated in our hospital from February 2019 to April 2021 were selected. The patients were randomly divided into the control group and the research group. The routine nursing mode was adopted in the control group, and the protective motivation intervention nursing mode was adopted in the research group. Nursing satisfaction, FIM score, Harris hip function score, WOMAC score, Barthel index score, and quality of life score were compared between the two groups.

**Results:**

The nursing satisfaction of the research group was higher than that of the control group, and there are statistically significant differences between the groups (*P* < 0.05). The FIM scores of the research group at discharge and 1 month, 3 months, and 6 months after discharge were significantly higher than those in the control group. The Harris hip function score of the research group was significantly higher than that of the control group at discharge and 1 month, 3 months, and 6 months after discharge. The WOMAC scores of the research group at discharge and 1 month, 3 months, and 6 months after discharge were significantly lower than those in the control group, and the difference was statistically significant (*P* < 0.05). The scores of the Barthel index at discharge and 1 month, 3 months, and 6 months after discharge in the research group were significantly higher than those in the control group. The scores of physiological function, psychological function, social function, and health self-cognition in the research group were significantly lower than those in the control group, and the difference was statistically significant (*P* < 0.05).

**Conclusion:**

The nursing model of protective motivation intervention for patients after hip arthroplasty can effectively improve the function of hip joint, improve the quality of life, promote the establishment of harmonious nurse-patient relationship, and play a positive role in improving the prognosis of patients.

## 1. Introduction

With the aggravation of the aging population in our country, the elderly are often accompanied by osteoporosis, cardiovascular and cerebrovascular diseases, diabetes, and so on, which are prone to be complicated with hip joint diseases such as femoral neck fracture and osteoarthritis [1–3]. At present, hip replacement has been quite mature, but the recovery of joint function of patients after operation is quite different. The reason is that, in addition to individual differences, most of them lack standardized and systematic training guidance for postoperative rehabilitation. Finally, it leads to poor recovery of joint function, and even some patients are in a state of depression, resulting in anxiety, resulting in the loss of social role and function [4, 5]. Protective motivation theory (PMT) is a widely accepted method, which is used as a general framework for predicting health behaviors and health-related interventions [6]. Protective motivation theory is one of the social cognitive theories used to evaluate protective behavior and factors affecting motivation and to explain effective and ineffective adaptive behavior when perceived health status is threatened [7]. The theory of protective motivation analyzes the emergence of healthy behavior from the perspective of motivational factors and discusses and explains the process of behavior change through threat assessment and coping assessment in individual cognitive regulation. At present, the theory of protective motivation is mainly used in the prediction and intervention of health behavior, and it has also been widely used in the self-management of chronic diseases. Domestic studies have applied this theory to chronic diseases and achieved good results [8]. Based on this, this study focuses on the effect of the protective motivation intervention nursing model on the functional recovery of patients after hip arthroplasty and its clinical significance.

## 2. Patients and Methods

### 2.1. Participant Information

Sixty patients who underwent hip arthroplasty in our hospital from February 2019 to April 2021 were selected. The patients were randomly divided into the control group and the research group. In the control group, the age was 43-74 years, with an average of 65.91 ± 3.63 years, including 18 males and 12 females, while in the research group, the age was 44-76 years, with an average of 65.96 ± 3.58 years, including 16 males and 14 females. There was no statistical significance in the general data of the two groups. This study was approved by the Medical Ethics Association of our hospital, and all patients signed informed consent.

The inclusion criteria were as follows: (1) age ≥ 18 years; (2) no cognitive, language, and intellectual impairment, with basic reading and writing ability; (3) patients who underwent hip arthroplasty for the first time; and (4) agreed to accept follow-up for 6 months and be able to accept and answer phone calls.

Exclusion criteria: (1) patients with severe heart, liver, renal insufficiency, malignant tumors, and other diseases; (2) patients who underwent hip replacement again; and (3) refusal to participate.

### 2.2. Nursing Methods

The control group received routine nursing intervention in the department, issued disease guidance manuals to patients on the day of admission, evaluated admission, patiently carried out health education for patients, and explained self-study points for attention to patients. For management after hip arthroplasty, individual nursing guidance was given, and health education was the main way of education.

On the basis of the control group, the research group implemented nursing intervention based on the theory of protective motivation, and the specific measures were as follows: (1) Understand the patient's problems and evaluate the needs: nurses communicate with patients one-on-one during the conversation. During this period, patients are free to ask questions and ask for help; when patients receive treatment or counseling, family members or others are allowed to accompany them. Start the dialogue with the following questions: how do you feel now (encourage patients to express their inner feelings)? Do you have any questions about this disease? How do you like to learn new knowledge? Through this needs assessment, nurses can understand which factors affect patients' learning and what knowledge patients already know and the defects of their knowledge or skills. It can provide a basis for working with patients to clarify learning priorities and learning opportunities. The nurse and the patient jointly explore the patient's understanding of the problem and work out a plan to respond and give the patient 5 minutes to ask the researcher, and the patient emphasizes the importance of joint decision-making between the patient and the health care person, to promote motivation and participation in behavior change. According to the preliminary assessment and patient goals, the researchers make a joint decision with the patients to make a plan, and on a regular and continuous basis, the researchers implement and adjust the nursing plan. (2) Health education: through the evaluation of patients' learning ability, it also provides patients with the opportunity to strengthen their understanding and master the skills to promote self-efficacy and self-management, through examination to ensure that patients can master disease-related information and practical skills. The first time (3 days after admission) content includes high risk factors, complications, and serious consequences of poor prognosis after hip arthroplasty. Its main purpose is to make patients aware of the consequences of untreated disease progression and related risks and complications and to increase their understanding of the severity and susceptibility of the disease. In the course of teaching, we can also introduce the bad cases of clinical patients' self-management to enhance patients' understanding of the serious consequences of bad lifestyle and promote their behavior change. The second time (5 days after admission) content includes individualized guidance to patients; basic knowledge of disease and drug treatment, including symptoms and course of disease, treatment strategies, and conventional disease control drugs; inviting caregivers to participate in the lecture; and strengthening family and social support, in order to reduce the external factors of self-management ability to improve the response efficiency of patients to take healthy behavior. The third time (1 week after admission) content includes conducting a demonstration to teach patients to master correct rehabilitation exercises, diet, and other skills, through antidemonstration teaching to ensure that patients have understood health information; researchers need to adjust their words according to the situation of patients, reduce the speed of speech, use less medical terms, and choose to use more straightforward language. In addition, nurses should strategically understand the patient's understanding and potentially wrong ideas to make sure that the patient's understanding is correct. (3) Peer support: lasted 1-2 hours, 6 patients at a time. Related studies have shown that the best group size for [9–11] patient experience exchange group meetings is designated as 6 to 10 patients, because this scale is large enough to minimize the impact of group learning but small enough for individuals to receive enough attention and support to ensure patient safety. Select patients with better disease control and higher disease self-management ability to be trained by senior nurses and head nurses, including life and medication guidance after hip arthroplasty. In the exchange meeting, they share their own experience and skills of self-management of disease, so that patients feel external rewards; that is, peers, families, and other external environment can promote the health behavior of patients, in order to promote the motivation and participation of patients' behavior change. In addition, the existing doubts were expressed among the patients, and the nurses encouraged the patients to express their confusion, so as to understand the environment and needs of the patients, and finally summarized and are guided by the medical staff. (4) Provide psychological care: carefully introduce the development of the disease and its prognostic treatment to patients and their family caregivers, so as to enhance their confidence in fighting the disease so that patients can actively cooperate with treatment and nursing. Nurses communicate personally to relieve patients' psychological pressure, improve their negative emotions as much as possible, and introduce successful cases to increase their hope of treatment. (5) Follow-up and individualized guidance: establish trust relationship with patients and their caregivers for the first time (2 weeks after leaving hospital); communicate with patients by telephone and WeChat to understand the problems existing in patients' self-management at the present stage. And set short-term goals for patients. For the second time (1 month after leaving hospital), the patients were revisited in the outpatient clinic to understand the current situation of disease control and self-management through communication and to evaluate whether the previously set short-term goals were achieved. Discuss with patients the problems existing in their behavior changes; make joint decisions between nurses and patients to find solutions; encourage caregivers to participate in the process of disease self-management, supervise, and promote the change of patients' behavior; and set long-term goals for patients. The patients were followed up for the third time (3 months after leaving hospital) to evaluate the implementation of patients' goals, complete the collection of questionnaires, analyze the problems existing in their self-management at the present stage, and jointly discuss the formulation of solutions. Ask patients for their evaluation and suggestions on the whole nursing intervention process.

### 2.3. Observation Index

#### 2.3.1. Satisfaction

After consulting the literature and experts' discussion, we designed patients' follow-up satisfaction [12], a total of 10 items, and recorded patients' satisfaction with follow-up management mode, health education, medical and nursing service, appointment registration process, and so on. It is divided into four dimensions: very satisfied, satisfied, general, and dissatisfied. Satisfaction rate = very satisfaction rate + satisfaction rate + general rate.

#### 2.3.2. FIM Scoring

Using the functional independent rating scale (FIM) [13], FIM was proposed by the American Association of Rehabilitation Medicine and the Society of Physical Medicine and Rehabilitation. It is a scale widely used to evaluate the daily activity ability of patients all over the world, including self-care ability, sphincter control, transfer, action ability, communication, and social cognition of five dimensions, a total of 18 items, the total score of 180.126; the higher the score, the better the functional independence of patients. The FIM scale has good intra- and intergroup reliability and good internal consistency.

#### 2.3.3. Harris Hip Joint Function Score

The Harris hip joint function score scale [14] is used to evaluate the therapeutic effect of hip joint disease, evaluated by medical staff, including pain, function, deformity, and range of motion of 4 dimensions, a total of 10 items, a total score of 100. The higher the score, the better the hip joint function.

#### 2.3.4. WOMAC Scoring

The Xi'an Osteoarthritis Index (WOMAC) and McMaster University Osteoarthritis Index (Osteoarthritis Index) [15] reflect the severity of joint injury and the recovery of joint function according to symptoms and signs, tend to be self-assessed by patients, and pay more attention to patients' subjective experience, including pain, stiffness, and joint function of three dimensions, a total of 24 items, the total score of 96; the higher the score, the more serious the joint damage. Cronbach's *α* coefficient of each dimension was 0.878-0.956, and the intragroup correlation coefficient was 0.82-0.88.

#### 2.3.5. Barthel Index

The ability of daily living (ADL) was evaluated by the Barthel index [16] before and after intervention, and the total score was 100. The higher the score, the stronger the ADL.

#### 2.3.6. Quality of Life Scale

The quality of life scale [17] includes four subscales of physical, psychological, social, and health self-awareness, with a total of 29 items. Cronbach's *α* coefficients of the scale ranged from 0.79 to 0.91. The scale was rated according to 1-5 grades. The lower the score, the higher the satisfaction.

### 2.4. Statistical Analysis

SPSS23.0 statistical software was adopted to process the data. The measurement data were presented as $\bar{x}\pm s$. The group design *t*-test was adopted for the comparison, and the analysis of variance was adopted for the comparison between multiple groups. The Dunnett *t*-test was adopted for comparison with the control group. The counting data were presented in the number of cases and the percentage, the *χ*^2^ test was adopted for comparison between groups, and the bilateral test was employed for all statistical tests.

## 3. Results

### 3.1. Comparison of Nursing Satisfaction

In comparison of nursing satisfaction between the two groups, the research group was very satisfied in 24 cases, satisfactory in 5 cases, and general in 1 case; the satisfaction rate was 100.00%, while in the control group, 14 cases were very satisfied, 10 cases were satisfied, 1 case was general, and 5 cases were not satisfied, and the satisfaction rate was 83.33%. The nursing satisfaction in the research group was higher than that in the control group, and the difference was statistically significant (*P* < 0.05). All the data are presented in Table 1.

### 3.2. FIM Score Comparison

Before nursing, there was no significant difference in FIM scores between the two groups, but after nursing, the FIM score of the two groups increased. The FIM score of the research group was higher than that of the control group at discharge, 1 month, 3 months, and 6 months, and the difference was statistically significant. All the data are presented in Table 2.

### 3.3. Harris Comparison of Hip Joint Function Score

Before nursing, there was no significant difference in the Harris hip function score between the two groups, but after nursing, the Harris hip function score of the two groups increased, and the Harris hip function score of the research group at discharge and 1 month, 3 months, and 6 months after discharge was higher than that of the control group, and the difference was statistically significant. All the data are presented in Table 3.

### 3.4. WOMAC Score Comparison

Before nursing, there was no significant difference in the WOMAC score between the two groups, but after nursing, the WOMAC score of the two groups decreased, and the WOMAC score of the research group at discharge and 1 month, 3 months, and 6 months after discharge was lower than that of the control group, and the difference was statistically significant (*P* < 0.05). All the data are presented in Table 4.

### 3.5. Barthel Index Score Comparison

There was no significant difference in the Barthel index score between the two groups before nursing, but after nursing, the Barthel index score of the two groups increased, and the Barthel index score of the research group at discharge and 1 month, 3 months, and 6 months after discharge was higher than that of the control group, and the difference was statistically significant (*P* < 0.05). All the data are presented in Table 5.

### 3.6. Comparison of Quality of Life Scores

There was no significant difference in the score of quality of life between the two groups before nursing (*P* > 0.05). The scores of physiological function, psychological function, social function, and health self-cognition in the research group were significantly lower than those in the control group, and the difference was statistically significant (*P* < 0.05). All the data are presented in Table 6.

## 4. Discussion

Artificial hip arthroplasty is an important method for the treatment of hip joint diseases in the elderly. Femoral neck fracture, osteoarthritis, osteonecrosis of the femoral head, and bone tumor are the most common indications. The purpose of the operation is to restore the function of the hip joint, improve the quality of life and quality of life of elderly patients, and help patients recover to their predisease state as much as possible [18]. With the development of orthopaedics, artificial hip arthroplasty has become the most effective method for the treatment of end-stage hip disease in the elderly, which is of great significance to improve the quality of life of elderly patients [19]. Rehabilitation training after hip arthroplasty is a gradual and long-term process, and patients can generally be discharged from the hospital and go home 2 weeks after operation, so more rehabilitation training needs to be completed at home [20]. However, most patients cannot get effective rehabilitation guidance after discharge, and most patients' discharge means the end of medical intervention, and there is a lack of rehabilitation training guidance after discharge. Due to care pressure, economic burden, lack of social role, and other factors, patients are prone to anxiety, irritability, lack of self-confidence, and other bad emotions, which are not conducive to postoperative recovery and patients' physical and mental health [21]. In the ever-changing complex medical environment, the original traditional expert education model has been transformed into the current patient participation model. In their own health decisions, patients become more active and responsible. In order to promote patients' self-management, patients have the right to have access to nursing information, tools, and other support related to them, so that they can actively participate in their own disease management [22]. Nurses are very important to patients' self-management. As nurses, we should promote patients' self-management in a way that patients can understand. The European Rheumatic Alliance emphasizes that patient health education is an integral part of standard care, and the purpose of health education is to encourage patients to participate in their own disease management in order to improve or maintain their quality of life [23]. Patient health education is considered to be a key part of the treatment of chronic diseases, and one of the roles of nurses is as health advocates; as the largest group of health care professionals, their role in providing team care for patients with rheumatic diseases follows the global trend of providing more proactive, evidence-based care for patients with chronic diseases [23, 24].

Protective motivation theory is developed by American scholars Ronald Dunn and Schwarze on the basis of health belief model theory and expectation theory in recent years [3]. Protective motivation theory holds that the formation of protective motivation is decision-making formed by people through threat assessment and response assessment [25]. Threat assessment is people's understanding of risk, which is formed after balancing the following two types of factors: one is to recognize the severity and vulnerability of risk factors, that is, the threat that risk factors may pose to their own interests; the other is the return after the implementation of risk factors, that is, the benefits brought by risk factors [26]. Among them, severity is people's judgment of the severity of the disease, including the response to the clinical and social consequences of the disease, and susceptibility is the subjective belief formed by people's subjective judgment of the possibility of suffering from a certain disease. It includes the individual's acceptance of the doctor's diagnosis and the judgment of the possibility of disease occurrence and recurrence [27]. Self-efficacy is people's confidence in the possibility that they can successfully take preventive actions and obtain the desired results. Response effectiveness and self-efficacy promote the occurrence of healthy behavior, while response cost reduces the possibility of healthy behavior. Individual threat assessment and response assessment work together to form protection motivation, which in turn promotes the occurrence or consistency of behavior. The internal return is the “benefit” that the individual perceives to take the risk factors, while the external return is the “benefit” that the individual perceives from the outside world. The severity and susceptibility of health threats are the factors to reduce adverse behavior reactions, and external and internal returns are the factors that promote the occurrence of adverse behavior reactions. Coping assessment is people's understanding of the ability to deal with health threats, and it is an assessment made after balancing the following two factors: one is response efficacy (RE) and self-efficacy (SE); the other is the response cost of implementing preventive actions (RC), that is, obstacles or inconveniences to take preventive measures, which is an obstacle that prevents people from taking certain actions or a reaction that affects protective behavior. Among them, response effectiveness is the understanding of the benefits brought by people after taking preventive measures [28, 29].

Combined with the results of this study, the comparison of nursing satisfaction between the two groups showed that the nursing satisfaction of the research group was higher than that of the control group, and after nursing, the FIM score, Harris hip function score, and Barthel index score of the research group at discharge and 1 month, 3 months, and 6 months after discharge were higher than those of the control group, while the WOMAC score was lower than that of the control group. In terms of the scores of quality of life, the scores of physiological function, psychological function, social function, and health self-cognition in the research group were lower than those in the control group. The analysis shows that when individuals are aware of serious health threats, susceptibility to diseases, low cost of behavior change, confidence and ability to change behavior, and less external returns for internal and bad behavior and think that behavior change is beneficial, it indicates that individual protection motivation is maximized and individual protection behavior is promoted [30, 31]. This study still has some shortcomings. Firstly, the quality of this study is limited due to the small sample size we included in the study. Secondly, this research is a single-center study, and our findings are subject to some degree of bias. Therefore, our results may differ from those of large-scale multicenter studies from other academic institutes. This research is still clinically significant, and further in-depth investigations will be carried out in the future. We followed the methods of other scholars [32–34], who have applied new methods to help doctors make accurate decisions in the diagnosis of heart disease.

In conclusion, the nursing model of protective motivation intervention for patients after hip arthroplasty can effectively improve the function of the hip joint, improve the quality of life, promote the establishment of a harmonious nurse-patient relationship, and play a positive role in improving the prognosis of patients.16386.7

## Figures and Tables

**Table 1:** Comparison of nursing satisfaction between the two groups (*n*/%).

Grouping	*N*	Very satisfied	Satisfied	General	Not satisfied	Satisfaction rate
Control group	30	14 (46.67)	10 (33.33)	1 (3.33)	5 (16.67)	25 (83.33)
Research group	30	24 (80.00)	5 (16.67)	1 (3.33)	0	30 (100.00)
*χ* ^2^						5.454
*P*						0.019

**Table 2:** Comparison of FIM scores between the two groups ($\bar{x}\pm s$, points).

Grouping	*N*	Before nursing	When discharged from the hospital	One month after discharge	Three months after discharge	Six months after discharge
Control group	30	97.83 ± 3.95	103.85 ± 3.85	108.35 ± 5.81	110.85 ± 3.95	118.84 ± 4.27
Research group	30	97.95 ± 3.41	115.93 ± 2.95	119.85 ± 1.84	123.82 ± 2.85	125.63 ± 3.95
*t* value		0.125	13.641	10.355	14.584	6.393
*P* value		0.900	0.000	0.000	0.000	0.000

**Table 3:** Comparison of Harris hip joint function score between the two groups ($\bar{x}\pm s$, points).

Grouping	*N*	Before nursing	When discharged from the hospital	One month after discharge	Three months after discharge	Six months after discharge
Control group	30	56.82 ± 4.91	60.86 ± 3.64	68.93 ± 4.91	75.91 ± 3.91	80.75 ± 3.95
Research group	30	56.91 ± 4.75	65.91 ± 3.91	78.72 ± 2.97	86.91 ± 3.95	90.83 ± 3.42
*t* value		0.072	5.177	9.344	10.840	10.566
*P* value		0.942	0.000	0.000	0.000	0.000

**Table 4:** Comparison of WOMAC scores between the two groups ($\bar{x}\pm s$, points).

Grouping	*N*	Before nursing	When discharged from the hospital	One month after discharge	Three months after discharge	Six months after discharge
Control group	30	45.95 ± 3.94	40.96 ± 3.91	35.76 ± 3.96	30.71 ± 3.91	23.86 ± 4.96
Research group	30	45.81 ± 3.91	36.85 ± 2.91	30.91 ± 2.93	26.76 ± 3.58	17.85 ± 3.92
*t* value		0.138	4.618	5.392	4.081	5.206
*P* value		0.890	0.000	0.000	0.000	0.000

**Table 5:** Comparison of Barthel index scores between the two groups ($\bar{x}\pm s$, points).

Grouping	*N*	Before nursing	When discharged from the hospital	One month after discharge	Three months after discharge	Six months after discharge
Control group	30	33.86 ± 3.91	46.91 ± 3.65	54.86 ± 5.64	78.83 ± 4.93	88.61 ± 3.84
Research group	30	33.75 ± 3.42	58.76 ± 4.71	65.86 ± 3.23	84.76 ± 5.74	98.71 ± 4.75
*t* value		0.115	10.892	9.269	4.292	9.056
*P* value		0.908	0.000	0.000	0.000	0.000

**Table 6:** Comparison of quality of life scores between the two groups before treatment ($\bar{x}\pm s$, points).

Grouping	*N*	Physiological function		Psychological function		Social function		Healthy self-cognition	
		Before nursing	After nursing	Before nursing	After nursing	Before nursing	After nursing	Before nursing	After nursing
Control group	30	15.84 ± 4.91	13.86 ± 2.95^a^	16.94 ± 3.91	14.85 ± 4.86^a^	18.82 ± 3.95	16.37 ± 2.81^a^	15.98 ± 3.91	13.86 ± 1.85^a^
Research group	30	15.96 ± 4.52	11.84 ± 2.91^b^	16.95 ± 3.86	12.81 ± 1.85^b^	18.84 ± 3.55	12.84 ± 3.81^b^	15.87 ± 3.66	10.83 ± 2.91^b^
*t* value		0.098	2.670	0.009	2.148	0.020	4.084	0.112	4.812
*P* value		0.921	0.009	0.992	0.035	0.983	0.000	0.910	0.000

Note: the control group before and after nursing, ^a^*P* < 0.05; the research group before and after nursing, ^b^*P* < 0.05.

## Data Availability

The datasets used and analyzed during the current study are available from the corresponding author upon reasonable request.
